This article has been retracted.

# Health Informatics on Adolescents Smoking Based on the Miryoku Engineering Analysis Framework

**DOI:** 10.1155/2021/8569273

**Published:** 2021-11-28

**Authors:** Jia-Xuan Han, Kun Wang

**Affiliations:** ^1^Pan Tianshou College of Architecture, Arts and Design, Ningbo University, Ningbo 315211, China; ^2^Institute of Fine Arts and Design, Quanzhou Normal University, Quanzhou 362000, China

## Abstract

Smoking among young people has aroused widespread concern in society. The number of young people who smoke has increased year by year, which has largely affected their health. Therefore, how to improve the prevention and control rate of tobacco harm, thereby reducing the smoking rate of young people has become an important issue. Based on the glamour engineering research method that can specifically solve the problem of attractiveness between users and products, the user preference of young people's smoking behavior is studied through the evaluation structure method and quantitative type I analysis, and the potential attractive factors are analyzed. Among them, there are 7 important attractive characteristics that affect the first attempt to smoke. These seven factors are divided into two aspects, namely, personal preference factors and environmental factors. The statistical data obtained through data analysis will be tested in the KMO field. The KMO values are 0.827 and 0.687, respectively, and the statistical results have obvious scores, so this study is effective. By quantifying one category, the partial correlation coefficients of different categories can be found, that is, specific solutions. This method provides a reference for ways and means to curb smoking behavior and also provides a case study for studying user perception. According to the research results, we seek ways to influence the smoking preferences of young people and then adopt some artificial methods to intervene in the generation of these factors, so as to achieve the purpose of reducing smoking among young people.

## 1. Introduction

The harm of tobacco to health has become one of the most serious public health problems in the world [1]. Note that 60% of smokers started smoking in their teenage years [2]. Therefore, reducing the smoking rate of adolescents is the key to reducing the overall smoking rate [3]. Youth tobacco control is of decisive significance to the entire tobacco control work. Pollution caused by smoking and second-hand smoke is the main factor affecting the health of young people. Therefore, how to effectively prevent and control youth smoking, reduce youth smoking rate, and protect youth health is an urgent task for public medical service providers. Although smokers know that smoking is harmful to the human body, they cannot resist the dependence and habit of smoking [4]. This is because it is difficult to quit the dependence caused by long-term smoking, but the interest in smoking in the early stage of smoking is not this dependence but is caused by other factors [5]. This shows that smoking habits are attractive to smokers. In addition to the physiological level of addiction, other psychological factors are rarely studied, especially during smoking behavior. Therefore, understanding the incentives of adolescent smoking from a psychological perspective can provide another reference level for preliminary prevention and control of smoking damage, which is of great significance. A prospective study of 4134 adolescents showed that smoking or exposure to second-hand smoke increases the risk of chronic cough and chronic bronchitis [6, 7]. The prevention and control of tobacco harm should be the highest education focus of schools and communities [8]. Tobacco control is globally recognized as the most effective measure to prevent and control a single risk factor. Therefore, how to formulate more targeted and effective strategic planning is particularly important.

Existing research on adolescent smoking mainly focuses on medical health, smoking behaviors and attitudes, the impact of smoking on adolescents, and the complications of adolescent smoking [9]. Hanewinkel et al. discovered the peculiarities of the relationship between tobacco marketing and youth smoking and verified that the exposure of adolescents to cigarette advertisements under high exposure is related to the occurrence of adolescent smoking [10]. Research by Skinner et al. found that black adults are more likely to smoke than white adults. However, compared with white youth, the smoking rate of black youth is still lower, and the lower smoking rate of black adolescents may be due to clear guidelines for protecting parents from drug abuse and the consequences of obvious noncompliance with these guidelines [11]. Leatherdale believes that the density of tobacco retailers around the school is related to the smoking behavior of students [12]. A questionnaire survey was conducted among 6967 7th grade students to evaluate smoking habits and smoking-related variables. The analysis shows that the best predictor of cigarette trials is that people can smoke easily and whether they smoke regularly seems to be affected by cost; the analysis also shows that variables related to weight are closely related to frequent smoking [13]. But most research is to control smoking behavior. How to control smoking for the first time is the key to solving the problem. This research introduces the theory of Miryoku engineering, which can deeply explore the Miryoku factors in the process of smoking behavior, can more accurately capture user preferences, curb and reduce preference factors, and provide a positive reference for teenagers' inactive activities and guidance. This study mainly uses the evaluation structure method of the Miryoku project and quantitative type I indicators to extract and analyze the Miryoku factor of smoking, so as to capture the Miryoku factor that attracts users from the smoking factor and point out the direction to quit smoking and prevent minors from smoking.

## 2. Methods

### 2.1. Data Collection

We use in-depth interview methods to conduct the first stage of qualitative research. Since the United Nations defines adolescents as 15–24 years old, the subjects of the in-depth interviews are 25 adolescents aged 18–22 with smoking habits; their professions are all college students. There are 8 women and 17 men out of 25 women. In each interview, there is an interviewer, a sound recorder, and an interviewee. Interviewers and recorders are the two main researchers. Interviewers and recorders must be familiar with the purpose of the interview, process operations, and other details, and without interfering with the interviewee's understanding of the subject, they keep the interview and record work smoothly, record the content of the conversation, and make a record. The process of conducting an in-depth interview is as follows. (1) Through in-depth interviews, understand the factors (specific conditions and characteristics) of young people's attraction to smoking. (2) Through the KJ (Affinity Diagram) method, summarize and sort out adolescents' abstract concepts on the Miryoku of smoking (abstract value judgment). (3) Summarize Miryoku factors through related Miryoku engineering research methods.

### 2.2. Miryoku Engineering and Research Methods

Miryoku is a user's subjective preference, which is a manifestation derived from personal character and behavior. Ujigawa convened many scholars in 1991 to start the study of the “Miryoku engineering” [14, 15], with the goal of “creating attractive products, space technology, and knowledge.” The Miryoku factor proposed by the Miryoku project refers to the fact that user satisfaction can be greatly improved after possessing or enhancing the positive Miryoku factor [16]. According to this view, reducing or reducing certain positive attractiveness will weaken user satisfaction. The Miryoku project is a design concept based on consumer preferences, which enables designers and consumers to build a bridge of communication [6]. Its research can help designers understand user preferences more accurately and help products increase attractiveness [7]. The main research methods of Miryoku projects include evaluation structure method and quantitative type I.

### 2.3. Evaluation Structure

The evaluation grid method is a qualitative interview analysis method, usually used for Miryoku engineering research [17–19]. This method is an improvement of the method proposed by Japanese scholars and is a method of psychological cognition from objects to things [20, 21]. This method is mainly to compare Subject A and Subject B through personal interviews to clearly discuss the similarities and differences between the subjects and sort out the various attributes of the subjects. Junaihiro Sanai (1986) divides Miryoku engineering's research method into two steps. The first step is to evaluate the target and answer the “pros and cons” or “likes and dislikes” of the target. The second step is to clarify the meaning of the answers through other questions and summarize the answers of the interviewees to specifically analyze the attractiveness factors of the product according to the preferences of users. After that, you can find the abstract reasons (higher: abstract value judgment), original evaluation items (median: perceptual perception), and specific constituent conditions (lower: objective and specific understanding). We rank specific things in the personal evaluation structure. This research method is called the evaluation grid method. The evaluation structure method is to conduct interviews from the perspective of comparing the “likes” of the evaluation objects. Respondents asked about the characteristics of the original evaluation items and objectives, then layered the mechanism of consumer evaluation through ladder diagrams, and asked about the abstract concepts and specific conditions and characteristics of the evaluation items. Repeated tasks can sort out the three levels of abstract concepts (higher position: abstract value judgment), original evaluation items (median position: object Miryoku characteristics), and specific constituent conditions (lower position: objective and concrete understanding). Then, we sort out the interview author's personal evaluation structure of specific things. Wang et al. proposed a method for evaluating the attractiveness of products based on Miryoku engineering through the case of electric kettles. The first is to identify the product form attractive factors. Then, Conjoint Analysis was employed to obtain product form attractiveness to consumers. This method can help designers to grasp consumers' preferences to product form attractiveness and specify design objectives [22]. On this basis, many scholars have combined different research methods to improve the evaluation method in order to increase the accuracy of the evaluation.

### 2.4. Factor Analysis

Factor analysis is an attribute-based method [23]. Subjects must evaluate or judge each sample through the Richter scale or semantic difference method and use the measured data as input for factor analysis. The purpose of using factor analysis is to represent the original data structure with fewer dimensions and retain most of the information provided by the original data structure. Therefore, through factor analysis, we can know which factor is highly correlated with which variable, so as to understand the meaning of the factor and name it. Strictly speaking, principal component analysis and factor analysis use different methods to reduce the number of variables. Factor analysis is an interdependent analysis technique, which includes many techniques to reduce space (or size). Its main purpose is to represent most of the original data structure with fewer dimensions while retaining the original data. The factor analysis is as follows.

(1) Standardization of the original variable: for each element in the original variable *X*,
  (1) $$\begin{array}{c} x_{ij}^{\prime }=\frac{x_{ij}-{\bar{x}}_{i}}{S_{i}}\left(i=1,2,\ldots ,P,j=1,2,\ldots ,n\right). \end{array}$$
Among them, mean ${\bar{x}}_{i}=\left(1/n\right)\sum_{j=1}^{M}x_{ij}$, standard $S_{i}=\sqrt{\left(1/\left(n-1\right)\right)\sum_{j=1}^{M}{\left(x_{ij}-{\bar{x}}_{i}\right)}^{2}}$, *n* is the samples number deviation of *X*_*i*_, the average value of the processed matrix is 0, and the variance is 1.
(2) Correlation matrix calculation: the standardized covariance matrix of *X* is
  (2) $$\begin{array}{c} R=\left[\begin{array}{cccc} 1 & r12 & \cdots & r1P\\ r21 & 1 & \cdots & r2P\\ \vdots & \vdots & \; & \vdots \\ rP1 & rP2 & \cdots & 1 \end{array}\right]. \end{array}$$
(3) To determine the number of public factors in order to reasonably explain the variables studied, it is necessary to retain more important public factors and eliminate unimportant public factors. From the perspective of feature roots, usually, when the cumulative contribution rate corresponding to the current *M* feature roots ∑_*i*=1_^*M*^*λ*_*i*_/∑_*i*=1_^*P*^*λ*_*i*_ reaches 0.85 to 0.95, other feature roots can be ignored to determine the common factors *F*_1_, *F*_2_,…, *F*_M_.
(4) Determine the factor score. In the above steps, the variables are expressed as linear combinations of common factors. Since the common factor can more fully reflect the correlation between the original variables, the common factor can be expressed as a linear combination of the original variables. It is helpful to describe the characteristics of the research object, namely,
  (3) $$\begin{array}{c} F_{j}=\beta_{j1}X_{1}+\beta_{j2}X_{2}+\cdots +\beta_{jP}X_{P}\left(j=1,2,\cdots ,M\right). \end{array}$$
(5) Measure the common factor score of each sample. In terms of factors, the number of equations *M* is less than the number of variables *P*, so *β*_jP_ can be estimated in the sense of least squares to obtain factor scores.

### 2.5. Quantitative Analysis

Quantitative theory belongs to qualitative multiple regression analysis, which is a classification multiple regression analysis method [24, 25], which is often used in perception engineering. In order to find the approximate functional relationship between the variables and other qualitative item groups, multiple regression analysis is used to determine the intensity of each qualitative item's influence on the target variable. The quantitative theory is to study the relationship between a set of qualitative variables *X* (independent variables) and a set of quantitative variables *Y* (dependent variables), quantify qualitative variables into quantitative data (such as 0 and 1), and use multiple regression analysis to establish dependent variable *Y*. The prediction of *Y* as an observable random variable is affected by *P* nonrandom factors *X*_1_, *X*_2_,… *X*_P_ and random factor *ε* if Y and *X*_1_, *X*_2_,… *X*_*P*_ have the following linear relationship:

(4) $$\begin{array}{c} Y=\beta_{0}+\beta_{1}X_{1}+\beta_{2}X_{2}+\cdots +\beta_{p}X_{p}+\varepsilon . \end{array}$$

In the formula, *β*_0_, *β*_1_,…, *β*_*p*_ are *p* + 1 unknown parameters; *ε* is an unobservable random error. It is usually assumed that *ε* ∈ *N* (0, *σ*_2_), and the nonrandom expression is as follows:

(5) $$\begin{array}{c} E\left(Y\right)=\beta_{0}+\beta_{1}X_{1}+\beta_{2}X_{2}+\cdots +\beta_{p}X_{p}. \end{array}$$

Each qualitative variable item is composed of multiple categories, and it is assumed that all samples must be selected in each qualitative variable item, and only one category can be selected, which can simplify the establishment of the regression formula *Y* = ∑*βX* + *ε*. *Y* is the predicted value of the experiment (exclusiveness discussed in this study), *β* is the weight score of the category (for example, the importance of the category), *X* is different categories (for example, exclusive souvenirs, virtual characters), and *ε* is the random variable (for example, average exclusivity score). We use this method to predict the variability of external benchmark data and events. The greater the value of the partial correlation coefficient in the quantitative statistical result, the greater the degree of influence of the category on the target item, and the greater the value of the multiple (re)correlation coefficient in the statistical result.

## 3. Results

The research method of this study is divided into two parts, as shown in Figure 1.

The first part is qualitative research methods, which mainly focus on in-depth interviews. Interviews were conducted according to the evaluation structure method of the Miryoku item, and finally, 52 Miryoku evaluation factors with the Miryoku of smoking were screened out. Then, according to the KJ method, two main abstract concepts of smoking Miryoku are derived, namely, the abstract value judgment of smoking Miryoku. The second part is quantitative research methods. The results of the in-depth interview and KJ were used in a questionnaire survey using the Likert five-level scale. According to the results of factor analysis, the attractiveness evaluation factors of young smokers are reduced, and the seven main attractiveness characteristics of young smokers are finally sorted out. Based on the above experimental results, a structural diagram of the evaluation of the attractiveness of adolescent smoking was drawn. According to the results of the evaluation structure, five Likert scales were used to conduct a questionnaire survey, and based on type I quantitative analysis, the final calculated weight of youth smoking attraction was calculated. The results of qualitative data analysis are shown in Tables 1 and 2.

We summarized and screened out 51 attractive evaluation factors from in-depth interviews and divided them into two categories. The first category is the personal preference reasons for the attractiveness of smoking among young people. There are 29 reasons in total. Starting from the heart of adolescents, they are mainly personal factors that affect adolescent smoking. The other is the environmental factors that make young people attracted to smoking. There are 22 kinds of environmental factors, mainly environmental factors that affect youth smoking. Through factor analysis, this study combined the attractiveness factors (specific conditions and characteristics) of adolescent smoking and finally got the 7 most representative attractiveness characteristics of adolescent smoking (original evaluation item). The quantitative data analysis results are shown in Tables 3 and 4.

The KMO value is between 0 and 1. The closer the value is to 1, the higher the correlation of the variables and the more suitable for factor analysis. The closer the value is to 0, the lower the correlation of the variable and the less suitable for factor analysis. Its KMO index is 0.827, so this factor analysis is meaningful. Through the analysis of the personal preference and Miryoku factors of adolescent smoking, the evaluation factors of personal preference and Miryoku can be summarized into four main factors, including enhancement of personal Miryoku, curiosity, functional orientation, escape, and relaxation.

As shown in Table 4, the KMO index is 0.687; this factor analysis is meaningful. According to the analysis of the environmental factors (external factors) of adolescent smoking, the attractiveness assessment factors (external factors) produced by the environment can be summarized into three main factors, such as learning (active exposure), must smoke (passive exposure), and smoking will make me happy (other contact methods).

Due to the inconsistent dimensions of the in-depth interview project, in order to ensure that each factor has the same status in the analysis, we first use SPSS23.0 software normal standardization method to standardize the in-depth interview data (*Z*-score transformation) to obtain a new data table. Then, the KMO field test was conducted on the factor analysis of personal preference factors and the factor statistics of environmental factors. The KMO values were 0.827 and 0.687, respectively, and the statistical results scored significantly. Therefore, it is appropriate to use in-depth interview data for factor analysis. Through in-depth interviews, in terms of personal preferences, there are eight factors that can enhance personal Miryoku, curiosity and experimentation have eight factors, function-oriented factors have seven factors, and six avoidance and relaxation factors. There are 10 factors in the environment, 9 factors in the factors that must smoke, and 3 factors in the factors that make me happy. We use the maximum variance method to rotate the factors to obtain the rotated factor loading matrix. If the cumulative contribution rate of each column in the matrix exceeds 75%, the indicators are classified into one category, and there are 7 common factors in the two sets of problems. Through the above analysis, 7 common factors such as X1∼X7 can be obtained, and the dimensionality reduction of 51 original indicators has been achieved.

## 4. Discussion

Based on the above research results, a structure chart for the evaluation of youth smoking attractiveness was constructed. Based on the above experimental results, a structural diagram of the evaluation of youth smoking attractiveness is drawn, as shown in Figure 2. According to factor analysis, the seven attractive characteristics of adolescent smoking are the initial evaluation items. Summarizing the specific Miryoku factors of the influencing factors of adolescent smoking can finally be concluded to a higher level: the abstract value judgment of adolescent smoking is divided into personal preference factors and environmental generation factors. The median smoking Miryoku features include enhanced personal Miryoku, curiosity experimentation, functional orientation, escape and relaxation, learning behavior, must smoke, and smoking makes me happy. The lower level is the 51 alluring factors of smoking, that is, 51 specific conditions and factors. We build an evaluation structure chart based on this.

In this study, within the theoretical framework of an attractive engineering system, the correspondence between the factors that affect the attractiveness of adolescent smoking is explored through quantification. The 7 qualitative variable items (*X*1–*X*7) are composed of 51 categories *P*1–*P*29 and *E*1–*E*22, and assuming that all samples must be selected in each qualitative variable item, and only one category can be selected, the regression formula *Y* = ∑*βX* +*ε*. We calculate the score of each category and calculate the partial correlation coefficient between each category and the item. The degree of the project can be judged according to the weight of the correlation coefficient, and the final calculation is the quantification of personal influence factors and environmental factors. In the quantitative category, the partial correlation coefficient is the weight of the relationship between each factor and the whole, and the determination coefficient is the basis for the reliability of the statistical results. In the quantitative category, the predicted value of *R* = 0.00∼0.19 has a low correlation, the predicted value of 0.20∼0.39 has a correlation, the predicted value of 0.40∼0.69 has a strong correlation, and the predicted value of 0.70∼0.10 is very relevant. Quantitatively, we explain the data in Table 5, the expiration constant between personal preference factors and adolescent smoking is 0.806, the multiple correlation coefficient is 0.843, and the determination coefficient is 0.71. Enhancing self-Miryoku is an important Miryoku of adolescents' personal preference factors, and seeking self-identity is an important reason for enhancing self-Miryoku. Among the curiosity test factors, the most important reason for smoking is curiosity and sensory stimulation. Function-oriented smoking can help increase inspiration. Among the escape and relaxation factors, smoking is the most important reason for relaxation and maintenance of life.

We interpret the data in Table 6 quantitatively. The constant term of environmental factors and the attractiveness of adolescent smoking is 0.85, the multiple correlation coefficient is 0.697, and the coefficient of determination is 0.486. The type of learning (active contact) is an important charisma feature among the environmental factors of adolescents. Many smokers are important reasons for learning (active exposure). Under the pressure of being afraid of not making friends and wanting to win the care and recognition of classmates, this is an important reason for having to smoke (passive exposure). Smoking makes me happy (other ways of contact), and the most important reason is that smoking caused by the warmth at home makes me happy.

## 5. Conclusions

According to this study, there are many reasons why young people smoke, including not only physical and psychological personal factors but also external environmental factors, such as the growth environment and social needs. Because adolescents are in a critical period of physical development, mental shaping, and social adaptation, it is also a stage where psychological conflicts and emotional behavior problems are high. As they grow up, they accept a series of temptations from school, family, and society. Young people are looking for a way of self-expression in the process of self-growth. This may be the main source of personal factors that affect the attractiveness of smoking. There are internal reasons for adolescent smoking. Curiosity-driven (or satisfying curiosity) is usually considered to be the main internal psychological factor for adolescents to smoke for the first time. There is nothing wrong with young people being curious about smoking. In a general sense, we should not curb young people's curiosity about smoking. Instead, we should properly guide this curiosity through systematic and strict smoking prevention education, so that it can be sublimated into curiosity and avoid this situation. The deteriorating mutation is the curiosity of smoking. Due to the pressure of family, school, and society, some teenagers choose to smoke to relieve stress and ease their emotions and self-regulate through smoking. In terms of the attractive environment for young people to smoke, the most attractive feature is learning (active exposure). Teenagers are in the early stages of learning to understand society and will actively imitate behaviors that they believe are more attractive due to relatives and friends. The frequency of contact is the highest and therefore the most affected. At the same time, with the development of online information, the scope of influence of young people has also expanded to cyberspace. In terms of smoking obligatory (passive exposure), the pressure from social relations is affected by interpersonal communication, and smoking must be passive. Through the factors that affect the attractiveness of adolescent smoking problem, it can be concluded that if adolescents are in a social environment and show that smoking has a certain good psychological and social feedback on people, then adolescents will have a higher acceptance of smoking and therefore will think smoking is a good social life habit. This research can be provided to relevant health and education departments, starting with these factors that attract young people to smoke and thinking about this issue from another level, so as to improve the efficiency of smoking prevention and control, so as to reduce the smoking rate of young people.

## Figures and Tables

**Figure 1:** Method flow Miryoku.

**Figure 2:** Evaluation structure diagram of youth smoking attractiveness.

**Table 1:** Personal preference factors of youth smoking attractiveness.

Personal preference factors		
P1. Curious	P11. Like to collect cigarette boxes	P21. A sense of sustenance
P2. Relieve boredom	P12. Bored	P22. Smoking is very artistic
P3. Stress reliever	P13. Looking for self-identity	P23. Smoke tastes good
P4. Show off to others	P14. Smoking makes me confident	P24. Learn to smoke with boyfriend
P5. Lose weight	P15. Smoking fashion	P25. Smoking is hot
P6. Feel “handsome” or “shaped”	P16. Enjoy the moment	P26. What it's like to be an adult
P7. Refreshing	P17. No other hobbies except smoking	P27. Noticeable
P8. Relax	P18. Tobacco tastes more	P28. The body is still young and will not cause major harm
P9. Help increase inspiration	P19. Smoking will be a role model	P29. Feel irritating
P10. Think it's fun	P20. Want to feel light and light	

**Table 2:** Environmental factors contributing to the attractiveness of adolescent smoking.

Environmental factors		
E1. Roommate will give smoke	E9. Students supply cigarettes to each other	E17. People around participating in club activities are pumping
E2. Human pressure	E10. Family is not warm, smoking makes me happy	E18. Learn to father smoking
E3. Do as the locals do	E11. For social entertainment	E19. It does not make sense not to smoke
E4. Net celebrities smoke and feel good	E12. For social entertainment	E20. There are many smokers in the same generation
E5. Tobacco as a reward	E13. Want to win the care and recognition of classmates	E21. There will be peer pressure for fear of not making friends
E6. The idol smokes and wants to be like him	E14. It's fun to light a cigarette for the family	E22. Neighbor taught me to smoke
E7. I heard family members talk about the benefits of smoking	E15. Influence of gangs, feel safe while studying	
E8. I cannot say no because of my classmate's invitation	E16. People around you treat, but I'm sorry to refuse	

**Table 3:** Factor analysis of personal preference factors (internal factors).

Component							
Item	Enhance personal charm	Item	Curious to try	Item	Function-oriented	Item	Escape and relax
P6.	0.896	P1.	0.961	P9.	0.779	P3.	0.906
P13.	0.808	P16.	0.833	P5.	0.688	P7.	0.895
P25.	0.771	P10.	0.806	P12.	0.673	P8.	0.845
P14.	0.73	P29.	0.788	P17.	0.624	P2.	0.747
P15.	0.727	P23.	0.737	P28.	0.605	P21.	0.687
P22.	0.690	P24.	0.726	P11.	0.587	P20.	0.670
P27.	0.623	P18.	0.603	P19.	0.544		
P4.	0.597	P26.	0.566				

**Table 4:** Factor analysis of environmental factors (external factors)

Component					
Item	Learn something	Item	Have to smoke	Item	Smoking makes me happy
E18.	0.854	E21.	0.706	E10.	0.576
E14.	0.844	E15.	0.688	E9.	0.535
E7.	0.721	E11.	0.637	E5.	0.527
E20.	0.687	E8.	0.626		
E1.	0.627	E2.	0.603		
E22.	0.595	E16.	0.596		
E17.	0.573	E13.	0.57		
E6.	0.557	E19.	0.533		
E4.	0.557	E3.	0.520		
E12.	0.551				

**Table 5:** Quantification of “personal preference factors” of youth smoking Miryoku type I results.

Item	Category points	Item	Category points	Item	Category points	Item	Category points
X1 enhance personal Miryoku	P6: −0.930	X2 curious to try	P1: 1.29	X3 function-oriented	P9: 0.38	X4 escape and relax	P3: 0.193
	P13: 0.813		P16: −1.73		P5: 0.12		P7: 0.133
	P25: 0.721		P10: −2.60		P12: 0.126		P8: 0.230
	P14: −1.015		P29: 0.82		P17: −0.12		P2: −0.023
	P15: −1.465		P23: 0.39		P28: 0.143		P21: 0.220
	P22: 0.660		P24: −0.07		P11: −0.006		P20: −0.071
	P27: 0.649		P18: −2.07		P19: −0.190		
	P4: −1.338		P26: −0.41				

Partial correlation coefficient	0.632	Partial correlation coefficient	0.818	Partial correlation coefficient	0.306	Partial correlation coefficient	0.459

**Table 6:** Quantitative type I results of “environmental production” of youth smoking Miryoku.

Item	Category points	Item	Category points	Item	Category points
X1. Learn something (valid contact)	E18: 0.580	X2. Have to smoke (passive contact)	E21: 0.312	X3. Smoking makes Me happy (other forms of contact)	E10: 0.268
	E14: 0.024		E15: 0.231		E9: 0.072
	E7: −1.582		E11: 0.026		E5: 0.058
	E20: 0.557		E8: −0.021		
	E1: −0.866		E2: 0.233		
	E22: −0.906		E16: −0.055		
	E17: −0.538		E13: 0.28		
	E6: 0.145		E19: 0.12		
	E4: −0.081		E3: 0.226		
	E12: 0.054				

Partial correlation coefficient	0.472	Partial correlation coefficient	0.558	Partial correlation coefficient	0.321

## Data Availability

The datasets and codes of this paper for the simulation are available from the corresponding author upon request.
